The article "Illuminating an Ecological Blackbox: Using High Throughput Sequencing to Characterize the Plant Virome Across Scales" was published in 2020. Journal: Front Microbiol.

# Illuminating an Ecological Blackbox: Using High Throughput Sequencing to Characterize the Plant Virome Across Scales

**DOI:** 10.3389/fmicb.2020.578064

**Published:** 2020-10-16

**Authors:** François Maclot, Thierry Candresse, Denis Filloux, Carolyn M. Malmstrom, Philippe Roumagnac, René van der Vlugt, Sébastien Massart

**Affiliations:** ^1^Plant Pathology Laboratory, Terra-Gembloux Agro-Bio Tech, Liège University, Gembloux, Belgium; ^2^Univ. Bordeaux, INRAE, UMR BFP, Villenave d’Ornon, France; ^3^CIRAD, BGPI, Montpellier, France; ^4^BGPI, INRAE, CIRAD, Institut Agro, Montpellier University, Montpellier, France; ^5^Department of Plant Biology and Graduate Program in Ecology, Evolution and Behavior, Michigan State University, East Lansing, MI, United States; ^6^Laboratory of Virology, Wageningen University and Research Centre (WUR-PRI), Wageningen, Netherlands

**Keywords:** virus ecology and evolution, plant virome, high throughput sequencing, historical advances, opportunities and challenges

## Abstract

The ecology of plant viruses began to be explored at the end of the 19th century. Since then, major advances have revealed mechanisms of virus-host-vector interactions in various environments. These advances have been accelerated by new technlogies for virus detection and characterization, most recently including high throughput sequencing (HTS). HTS allows investigators, for the first time, to characterize all or nearly all viruses in a sample without *a priori* information about which viruses might be present. This powerful approach has spurred new investigation of the viral metagenome (virome). The rich virome datasets accumulated illuminate important ecological phenomena such as virus spread among host reservoirs (wild and domestic), effects of ecosystem simplification caused by human activities (and agriculture) on the biodiversity and the emergence of new viruses in crops. To be effective, however, HTS-based virome studies must successfully navigate challenges and pitfalls at each procedural step, from plant sampling to library preparation and bioinformatic analyses. This review summarizes major advances in plant virus ecology associated with technological developments, and then presents important considerations and best practices for HTS use in virome studies.

## Introduction

The field of plant virus ecology examines complex interactions among plant-associated viruses, their hosts and their vectors, and the environment, effectively extending the perspective of plant virus epidemiology (Jones, 2014). Traditionally, virus epidemiology investigates diseases and factors influencing their spread and population dynamics, whereas virus ecology extends the focus to include understanding patterns of virus distribution and dynamics within a given environment, their effects on community and ecosystem properties, and the reciprocal effects of the environment on virus dynamics and evolution (Gibbs, 1983; Hull, 2014; Lefeuvre et al., 2019).

As a field, plant virus ecology draws on diverse disciplines including virology, ecology, epidemiology, plant biology and entomology (Matthews and Hull, 2002). The study of viruses requires highly specialized methods and tools, which explains why at first ecologists focused their efforts on more readily observable organisms and why the history of plant virus ecology has largely been driven by technological developments (see Figure 1). Plant virus ecology has also been marked by the gradual divergence of virology and ecology during the 20th century, caused by the development of molecular methods from the 1970s onward, which oriented virology toward virus molecular biology and the study of viral infection in controlled conditions, away from ecological considerations (Malmstrom et al., 2011). This gap between the fields of ecology – mainly focused on wild and less managed ecosystems – and virology, centered on model or domesticated hosts, began to be bridged in the early 21st century by the use of new genomic tools and molecular approaches in ecological studies (Malmstrom et al., 2011). Most of these new tools involve High-Throughput Sequencing (HTS) technologies, also called Next Generation Sequencing (NGS). Taken together, these developments have spurred the emergence of plant virus metagenome studies. The metagenome, or “virome” when referencing viruses, corresponds to the collective genome of a microbial community within a given individual or a defined environment (Roossinck, 2012). Studying the plant virome in natural communities is currently strongly advancing knowledge of viral diversity, identifying new viral variants or species that might emerge in the future as significant pathogens, and identifying new hosts of known viruses (Roossinck et al., 2015; Massart et al., 2017). Going forward, a better understanding is needed for many aspects of virus ecology: reservoirs, exchange among hosts in various landscapes, lifestyles of plant viruses, contribution of viruses to the functioning of plant populations and communities, the impact of agricultural practices on viral populations, etc.

**FIGURE 1:** Time line of the major advances in plant virus ecology, linked to the evolution of the detection methods.

We describe here the evolution of the techniques used in plant virus ecology and their respective impact in this field, emphasizing new high-throughput sequencing-based approaches. Several reviews have already been published on virus ecology and HTS (Roossinck, 2012; Roossinck et al., 2015; Stobbe and Roossinck, 2014) but as of yet none has detailed the opportunities and the technical challenges of applying HTS technologies with a plant virus ecology perspective. The chronology of the major advances in plant virus ecology, as well as the technological developments supporting them, is represented in the historical timeline of Figure 1.

## Early Stages of Plant Virology and of Plant Virus Ecology

The first plant virus infection phenotypes were likely recorded more than 1,200 years ago in *Eupatorium* plants in Japan in AD 752, as highlighted by Saunders et al. (2003). But the early stages of plant virology were marked by the description of the first plant virus, tobacco mosaic virus (TMV), by concomitant studies of Mayer (1886), Beijerinck (1899), and Ivanovskij (1899) at the end of the 19th century, using the observation of symptoms on tobacco plants.

Since the discovery of TMV, scientists have sought to study the interactions between plants and viruses, but also to decipher how viruses are transmitted between plants. Hence, the first half of the 20th century saw the building of the foundations for plant virus ecology, thanks to the use of host symptomatology, sap transmission, indicator plants, biochemistry and microscopy (reviewed in Harrison, 2009). The first explorations of plant-virus interactions involved cultivated plants and led to important insights, such as the existence of asymptomatic infections (Nishimura, 1918) or of multiple infections (Dickson, 1925). In the 1930s plant virologists began to show interest in wild communities. Brief surveys on wild plants, carried out in Germany in 1932–33 and in England in 1948–49, revealed high rates of viral infections in weeds, and a longer-term study was implemented between 1951 and 1954 in order to determine the frequency and distribution of plant viruses in their natural environment (MacClement and Richards, 1956). Virus flow between wild and cultivated reservoirs was demonstrated (Storey and McClean, 1930), as well as asymptomatic viral infections in many wild plants (Bennett, 1944).

In parallel, virologists examined interactions between viruses and their vectors, illustrated by the discovery of the first insect vector of plant viruses in 1901 (Takami, 1901). The importance of insects in virus transmission brought the concept of the “ecological trinity” between viruses, their hosts and their vectors, as coined by Carter (1939). The relationships between insect-borne viruses and their vectors led to the notions of “persistence” or “non-persistence” according to the period over which the vector can transmit the virus following its acquisition (Carter, 1939). Other virus vectors were identified, such as fungi [*Olpidium* spp. for lettuce big vein virus, (Campbell, 1962)] and nematodes [*Xiphinema* spp. for grapevine fanleaf virus, (Hewitt et al., 1958)]. Interactions between viruses themselves were also examined, leading to the discovery of synergisms (Vanterpool, 1926; Bennett, 1944) and antagonisms between virus strains or species (Bawden and Kassanis, 1941, 1945). Finally, early stages of plant-virus-vectors interactions were illustrated in 1951 with the demonstration that a virus can manipulate its host plant and vector, through a differential effect on aphids feeding on healthy or infected plants (Kennedy, 1951).

## The Development of Molecular Tools

The rise of serological and molecular detection tools was a golden era for the discovery of the vectors of plant viruses. Indeed, plant viruses were found to be transmitted by a wide range of agents, especially sap-sucking insects (e.g., aphids, thrips, whiteflies, leafhoppers), but also by beetles, mites, nematodes, fungi, and protists. It was also revealed that plant viruses can be vertically transmitted *via* infected pollen or seeds (reviewed by Harrison, 1981 and recently in Lefeuvre et al., 2019). Screening of plant viruses in many plants and insects by the Polymerase Chain Reaction (PCR), Enzyme-Linked ImmunoSorbent Assay (ELISA), and radioactivity (dot blots, tissue printings, etc.) revealed that the host and vector ranges of some plant viruses are remarkably wide (Timian, 1974; Sherwood et al., 2003; Zitter and Murphy, 2009). This variability is also reported for virus transmission, with a great diversity in host ranges for given vectors (Wijkamp, 1995; Wilson, 2014). Despite this diversity of virus biological properties, many plant viruses studied to-date are considered as host generalists and vector specialists, i.e., they have a wide host range but a narrow range of vectors (Power and Flecker, 2003). Advances in deciphering routes of virus transmission were also made, in particular concerning the description of circulative and propagative transmission modes (Gildow, 1985; Ullman et al., 1993), and the concepts of phenotypic mixing or transencapsidation (Rochow, 1970). In parallel, advances in plant-virus interactions were made at the molecular level, with for instance the discovery of the role of helper component (Thornbury et al., 1985), the concept of RNA silencing of viral genes by the host and its viral suppression (Lindbo et al., 1993; Wang and Maule, 1995; Voinnet et al., 1999), or the role of genetic recombination in virus evolution (Bujarski and Kaesberg, 1986).

Major advances in understanding plant-virus co-evolution were obtained too, with the confirmation that virus infections could commonly be found in asymptomatic wild plants (Kelley, 1994; Creamer et al., 1996; Anaya-López et al., 2003). This was extended by the suggestion that some viruses could potentially be beneficial to plants (Gibbs, 1980; Xu et al., 2008). Overall, plant-virus interactions were shown to be complex and to vary along an antagonism-mutualism continuum according to host and virus genotypes combinations and to environmental conditions (Gibbs, 1980, reviewed in Fraile and García-Arenal, 2016). In addition, co-infections with several viruses were frequently found in crops and in wild plants, further increasing the complexity of these interactions (Hammond, 1981; Jooste et al., 2015). Plant viruses were also found to be able to manipulate both their hosts and/or their vectors in order to maximize their transmission in plants (Mauck et al., 2010; Ingwell et al., 2012; Moreno-Delafuente et al., 2013), and reviewed in Mauck (2016).

## The Advent of Viromics

Studies of plant-virus interactions at the interface between managed and natural vegetation have been conducted for nearly a century (as reviewed in Alexander et al., 2014) but became more common in the 21st century, facilitated by PCR and new sequencing techniques, most recently HTS. HTS-based metagenomic studies were initially mostly performed to explore plant virus diversity, demonstrating it to be largely underestimated (Roossinck et al., 2015; Wren et al., 2006). Plant virus-like nucleic acids were further detected in many environments [(Culley et al., 2006; Kreuze et al., 2009) and reviewed in Roossinck, 2012; Roossinck et al., 2015], revealing an intriguing ability to circulate and persist with ecological implications that are not well understood. Viruses detected in metagenomic studies can be classified in four different types: (i) known viruses already described in the surveyed environment; (ii) known viruses not previously described in the surveyed environment; (iii) new virus species/isolates from a known family, and (iv) totally new viruses (Stobbe and Roossinck, 2014). This diversity of known/unknown plant viruses using metagenomic studies was first identified from pooled samples, further probed in analyses of individual barcoded plants [ecogenomics studies (Roossinck et al., 2010)], and then considered in an explicit spatial context [geometagenomic studies (Elena et al., 2014; Roossinck et al., 2015)].

Up to now, most HTS studies have been focused on virus identification and characterization in cultivated plants (Stobbe and Roossinck, 2014). In contrast, metagenomic studies on wild plants have been scarcer (Stobbe and Roossinck, 2014), but have confirmed that virus infections are common in nature (Muthukumar et al., 2009; Claverie et al., 2018, 2019; Susi et al., 2019) and may not cause any recognizable symptoms in wild plants in natural settings. These studies further reveal an abundance of persistent viruses (i.e., viruses that do not move between cells in plants but are transmitted in a strictly vertical manner via gametes) (Roossinck, 2010). The central value of these studies in expanding our understanding of viral diversity has been well-recognized. Indeed, a recent taxonomic position paper recommended the incorporation of viruses identified only from metagenomic data into the official classification scheme of the International Committee on Virus Taxonomy [ICTV, (Simmonds et al., 2017)], in parallel with the development of robust frameworks and safeguards for sequence-based virus taxonomy. Major discoveries in metaviromics and viral phylogenomics have caused conceptual shifts in plant virus evolution and ecology, recognition of the influence of co-divergence, host switching, and horizontal virus transfer (HVT) from invertebrates and fungi, on the origins and diversification of the plant virome (Shi et al., 2016; Zhang et al., 2019; Dolja et al., 2020). These discoveries redefined the RNA virosphere and virus evolution pathways, and enable development of the first comprehensive virus megataxonomy (Koonin et al., 2020).

Metagenomics-based inventories of plant viruses can inform significant current issues in virus ecology, including the emergence of new virus diseases, the impact of climate change or of anthropic pressures on viral populations and on plant-virus-vector interactions, the contribution of plant viruses to the functioning of wild plant populations, rules driving the assembly of viral communities etc. (as reviewed in Jones, 2014). Consequently, molecular and recent HTS-based studies have advanced our understanding of several important phenomena: (i) the reciprocal influences between the dynamics of pathogens and the structure of multispecies host communities (Power and Mitchell, 2004), illustrated with invasions of non-native plants (Malmstrom et al., 2005; Borer et al., 2007); (ii) plant virus spread among host reservoirs (wild and domestic) (Ma et al., 2020); (iii) spill-over and spill-back events (Elena et al., 2014; Roossinck and García-Arenal, 2015); (iv) effects of ecosystem simplification caused by human activities (and especially agriculture) on the biodiversity and the emergence of new viruses in crops (Pagán et al., 2012; Bernardo et al., 2018; Alonso et al., 2019, reviewed in Roossinck and García-Arenal, 2015; McLeish et al., 2019); and finally (v) effects of host diversity and genetic heterogeneity on virus dynamics (Power, 1991).

## Plant Virus Ecology and HTS: Opportunities

The ability of HTS technologies to potentially detect, without *a priori* information, all or nearly all viruses within a sample offers a huge opportunity to improve virome characterization and supports the study of virus richness at multiple scales, from individual plants to entire ecosystems. In addition, these technologies also provide new insight about deciphering intra-specific viral diversity, facilitating the characterization of virus variants and better disentangling viral population genetics. In the future, HTS might also be used to quantify the relative proportions of virus species and variants within a sample or environment, thus permitting new analyses of virus prevalence and co-infection dynamics.

HTS technologies have significantly accelerated the discovery of novel viruses and of new wild hosts for known viruses. In many cases, HTS provides a strong advantage for virome characterization over the application of a large number of specific ELISA or (RT-) PCR detection protocols (Boonham et al., 2014; Massart et al., 2014), in particular when taking into account novel viruses. If the aim is to independently characterize the virome of multiple plant species within a community, the number of potentially targetable viruses becomes even greater, making targeted detection approaches more complex if not unrealistic. This fact – and the cost of large targeted efforts – explains in part why virus ecological studies have so far largely focused on a small number of virus species. Thanks to its untargeted and comprehensive approach, HTS has the potential to allow more comprehensive studies of the plant virome at community and landscape scales (Prabha et al., 2013).

Bioinformatic advances leverage the power of HTS technologies and provide further insight about viral genomes. Given sufficient sequencing depth or target availability, contigs assembled from short reads (e.g., from Illumina^TM^ sequencing) or native long-reads (e.g., from Nanopore^TM^) can potentially represent the full or nearly full genome of a virus.

## Plant Virus Ecology and HTS: Challenges

HTS technologies can provide a comprehensive analysis of the viruses and variants present within a sample, and allow their detection, sequence characterization and, potentially in the future, relative quantification. Nevertheless, HTS application in plant virus ecology may be hindered by challenges that limit the sensitivity and/or specificity of species/variant detection and their relative quantification (see Figure 2). Until recently, HTS technologies have been widely used on single plants to discover new viruses or strains or to study viral population genetics within individual plants. A current issue is to ensure smooth and smart transition from sequencing individual plants to large plant populations. The central challenge is that whereas low cost (RT-)PCR and ELISA tests can be carried out on large numbers of individual plants, the high per sample cost of HTS technologies often requires balancing sequencing depth/cost with the number of plants analyzed, for example by the pooling of plant samples. This pooling step has consequences for the interpretation of results. Thus, the transition to work at broader scales raises a series of issues that must be surmounted. Here we consider these issues in more detail.

**FIGURE 2:** Methods for characterizing the viromes of plant communities. Various factors may potentially impact HTS-based viral ecology studies, at the different steps of these studies: plant sampling at days post-infection (DPI), field sampling, pooling strategies, sample and library preparation methods, selection of the sequencing platforms and bioinformatic analyses. Biological data on the viruses, their host plants and vectors (if known) could also be useful for viral ecology studies.

### Selection of Plant Sampling Strategy

Depending on the research aim – which might be the study of a single virus or of holistic virome diversity – there are several possible plant sampling strategies, including one-time and repeated measures. For one-time sampling, the crucial point is to determine the optimal sampling date in relation to the research objectives, perhaps when virus titers are highest (see below), at periods of greatest viral diversity, or after a certain period of virus spread, etc. For virome diversity studies, the lack of information makes it very complicated (perhaps impossible) to determine the optimal sampling period for novel viruses. In that case, it may be best to use repeated sampling.

#### Virus Concentration (Titer)

Several factors influence the multiplication rate of viruses and their accumulation within plant hosts: the time of sampling, i.e., days post-infection (DPI); environmental conditions (Cordoba et al., 1991; Nachappa et al., 2016); phenological stage of the plant (Dal Zotto et al., 1999); sampled organ(s) (Kogovšek et al., 2011; Constable et al., 2012; Lacroix et al., 2016), and plant and virus genotypes (Azizi and Shams-bakhsh, 2014). The detection sensitivity for a single virus, as well as its genome coverage, depend on its concentration in the sample, on the sample processing method, and on sample sequencing depth (Visser et al., 2016). The genome of a low-titer virus is therefore less likely to be completely sequenced with good coverage, which will impose limits on population genetics studies.

There is generally no optimal sampling, but virus titers are typically higher in actively-growing, green vegetation than in senescent plant tissues. In-depth knowledge of biology of the known viruses within the plant community is therefore a bonus and should guide the choice of sampling time(s). For instance, temperate climate pathosystems involving aphids may be preferentially sampled in spring and autumn, when plants are growing actively and vector populations are expanding and actively disseminating (Harris and Maramorosch, 1977). This would therefore warrant sampling at multiple time points to provide a dynamic vision of the virome. If the budget is limited, a smart approach can be to first conduct large-scale screening by HTS followed by assessment of the kinetics of targeted virus prevalence by ELISA or (RT-)PCR.

#### Co-infection by Several Viruses

The broad application of HTS technologies for plant virus detection has driven a paradigm change: co-infections are now recognized to be much more frequent than single infections (reviewed in Mascia and Gallitelli, 2016). Such co-infections may have consequences for symptom expression and/or virus concentration, and therefore the probability of detection. Indeed, interactions of multiple viruses within a single plant or tissue can lead to a variety of relationships ranging from antagonism (Wintermantel et al., 2008; Tatineni et al., 2010; Syller and Grupa, 2014) to synergism (Wang et al., 2002; Martínez et al., 2013), depending on host, viruses involved and infection history (defined as the succession of infection events).

Co-infection may also cause competition among viral targets for sequencing reads; a low-titer virus could theoretically be missed in a co-infection if the other virus(es) have high titer. The presence of several strains or several viruses sharing regions of homology can also hamper the proper reconstruction of viral genomes. Indeed, around the homologous region (for which a single contig will be generated), several 5′ and 3′ flanking reads and contigs can be assembled, which can *in fine* produce chimeric assemblies. This issue has been demonstrated for closely related species most particularly, but not only, when using a small RNA sequencing protocol (Massart et al., 2019).

### Field Sampling

The protocol used for collection of samples from the field is critical but often poorly documented in virological reports. To support robust data analysis and interpretation, it is essential to consider the relationships among the question to be investigated, the overall study design, and the sampling strategy. Three common aims of field sampling for HTS studies are (i) to quantify *infection prevalence –* the proportion of individual plants that have detectable virus infection; (ii) to characterize the *species (or variant) composition* of a viral community or population; and (iii) to evaluate patterns of viral *diversity*, including viral *taxa richness* – the number of taxonomic units, such as species, genera, or families within a community. There are both general and aim-specific sampling considerations.

#### General Sampling Considerations

Many practical ecological and epidemiological texts offer guidance about field sampling strategies, including the classic “Measuring and Monitoring Plant Populations” (available online)^1^. Sampling insect communities raises additional considerations beyond the scope of this article. The interested reader is directed to specific literature on this question, in particular (Dayaram et al., 2015). Questions to consider include: What spatial pattern and areal extent of sampling will be the most suitable? What host species will be chosen? When and how frequently should sampling occur? How many individuals of each sampling group will be selected? What will be the specific process for plant selection – will developmental stage, size, or symptom status be considered? The answers to these questions will influence the nature of the statistical analyses that can be conducted and the inferences drawn.

In heterogeneous landscapes, planning may further involve discernment of plant community types within a larger sampling unit and development of a stratified sampling scheme in which sampling effort is allocated to each community type as a function of its relative area. If a larger unit is 40% dry meadow and 60% wet meadow, for example, sampling effort might be allocated proportionately.

Once sampling compartments are identified, protocols must be developed for determining (i) at which points material will be collected, and (ii) how much of each plant(s) will be collected at each point. Decisions about sampling locations are best made prior to entering the field to remove user bias. For example, pre-determined points can be selected in the lab with a Geographic Information System (GIS) and then located with a Global Positioning System (GPS) in the field. These points might be located completely randomly or be selected in a grid for systematic sampling (Bernardo et al., 2018). If a grid is used, care must be taken that the spacing does not align with a regular interval in the vegetation pattern that would lead to oversampling of some vegetation types and undersampling of others. Alternatively, sampling may be conducted at predetermined intervals along transects, an approach that requires less technology to implement (Wilson, 2014). One method is to walk along one or several transects within a community or landscape, collecting samples every certain number of paces (Sseruwagi et al., 2004; Turechek et al., 2010). Transect start points and headings may be selected randomly or deliberately chosen to capture particular features, such as distance from edge (Ingwell et al., 2017) or border communities containing alternative host species (Byamukama et al., 2011; Muñoz et al., 2014).

Once sampling points are chosen, it is also essential to develop a protocol guiding the selection of individual samples at each point. The sampling unit might be an individual plant, several plants, or a quadrat from which all or some of the plants are collected (Byamukama et al., 2011). A sample-selection protocol is necessary to prevent introduction of bias by the sampler whose eyes may be drawn, for example, to symptomatic plants (Wilson, 2014) or to larger ones. Selection may be made through a specific randomization process or selection pattern (e.g., the individual closest to the right of the point is sampled, irrespective of condition or size).

#### Infection Prevalence

Studies aimed at quantifying infection prevalence – a common objective in agricultural research – focus on determining the proportion of plants carrying infection. In this context, virus infection can be considered as a plant characteristic, and plants can be sampled using standard plant ecology methods. Individual plants may be barcoded separately and sequenced. Alternatively, pooled plants may be sequenced and then viruses of interest targeted in individual plants with specific (RT-)PCR or ELISA methods. A critical consideration is to ensure that individuals are sampled without regard to symptoms and that all age/size classes of interest are evaluated.

#### Virus Community Composition

A more complex aim is to characterize the virus community (“virome”) within a given area, plant community, or plant population. Typically, the objective is to identify all or most of the viral taxa within the study unit and perhaps also to compare virus community composition across host species, locations, or treatments. Important questions include, (i) Will the sampling protocol return a representative sample of the study unit? (ii) Can the desired comparisons across study units be fairly made?

To characterize the virome infecting a given plant community, the sampling effort may be structured to reflect the relative representation of the plant community’s members, as evident in their relative abundance, relative cover, or relative biomass. A virome reflecting the relative abundance of individual plant species could be achieved, for example, by complete random sampling of individual plants, given sufficient sampling effort. Alternatively, sampling that is representative of plant species’ relative abundances might also be achieved by first evaluating plant community composition and then conducting stratified sampling in which each plant species is sampled in proportion to its relative abundance. A third approach is to harvest all of the plants within numerous randomly-placed quadrats (often called the “lawn-mower” strategy) (Ramsell et al., 2008; Roossinck, 2012). This approach might be the most suited for analyses that aim to characterize an areal-based virome, but may also reflect to varying degrees the relative abundance, cover, or biomass of individual plant species. A critical issue for all methods is the extent of spatial dispersion or aggregation of samples, which will influence estimates of viral community composition and its comparability. For example, plants and viruses that are sampled in close proximity to each other are likely to be more similar than those with greater separation. Thus, samples taken from quadrats may miss species found in completely random sampling.

A related issue is the sampling effort – how many samples are to be taken overall? Typically, greater sampling effort uncovers greater species numbers, and the prevalence of individual viruses, as well as the relative representation of their plant hosts, will directly influence their probabilities of detection. If the prevalence or titer of a given virus is low, more sampling effort will be required to detect it, as it is also true for rare host species (Abarshi et al., 2010). *Taxon accumulation curves (collector’s curves*) illustrate the gain in species numbers detected with increasing sampling effort, but do not predict species identity. They are sometimes used, however, to roughly assess the sampling effort at which species number begins to saturate (Gotelli and Colwell, 2001).

In addition to capturing a representative plant community virome, some studies also seek to compare the viromes of individual plant species within it. This is straightforward if the relative abundances and samples of the plant taxa to be compared are similar. However, if one plant species is common and the other is rare, the sample size of the rare species in a community-representative sample may be too small to be effectively compared. For such comparisons, additional equal-numbers sampling of each plant species might be conducted, while keeping in mind that equal numbers will not represent equal proportions of the host populations. For example, 30 individuals might represent 80% of a rare population but only 1% of a common one. Thus, the virome of the rare host population will likely be more complete than that of the common host. For discussion of an alternative approach, standardizing to equal coverage, see Chao et al. (2014). To reduce sampling costs, the host-comparative and community–representative approaches might be combined by sampling all individual plant species in high numbers and then creating a community-representative assessment by subsampling each plant taxon in proportion to its relative abundance (this can be done multiple times to evaluate variability in outcomes). Such a combined approach is probably most tractable when barcoded plants are sequenced individually, because pooling steps in library preparation add complexity.

#### Virus Richness and Diversity

A third key aim of HTS studies is to evaluate patterns of *virus diversity*, as distinct from determining the taxonomic composition of the virome. Diversity is a core ecological property that can be complex to measure [for an introductory overview, see McCabe (2011)]; and further discussion in Gotelli and Colwell, 2001, 2011]. The simplest measure is *taxa richness* (*S*) or the number of different taxonomic units within a community sample. A related measure is *taxa density*, the number of taxonomic units per unit area. More complex indices, such as the Shannon-Wiener diversity index (*H’*) and Simpson’s diversity index (*D*_1_), incorporate information about both taxa richness and their relative abundance or evenness; the choice of index – of which there are many – may strongly influence the interpretation of results (Chao et al., 2014). Diversity is classically considered at several scales, as alpha, beta and gamma diversity. To simplify, alpha diversity describes diversity within a given subunit (sample, field, etc.), whereas beta diversity describes diversity among subunits or along environmental gradients. Gamma diversity represents diversity across an entire landscape, and incorporates both alpha- and beta- components (Whittaker, 1960).

In comparing diversity values, it is critical to consider equitability of sampling effort because the number of taxa discovered will increase with sampling intensity, as noted earlier. It is also important to note that sampling for diversity metrics may be either “individual-based” or “sample-based.” Individual-based assessments examine randomly chosen individuals in the field, whereas sample-based assessments evaluate the number and identity of the target taxa in collective sampling units such as quadrats (Gotelli and Colwell, 2001). Because of within-patch similarities, species richness values from sample-based assessments will generally be lower than equivalent individual-based assessments. When assessing viral diversity, essentially all measures will be sample-based, because viruses are not sampled directly as individuals standing independently in the field but rather as entities embedded within particular host environments, be they individual plants or multi-plant collections.

With regard to sampling effort, richness in the simplest example quantifies the number of taxa represented by a given number of enumerated individuals. For example, if one finds 100 individual viruses (virus counts, however defined) in each of two communities and this number represents 7 taxa in community A and 25 in community B, then viral taxa richness is much greater in community B, all else being equal. (In practice, richness values may be adjusted to account for differences in detection rates among species and other issues beyond the scope of this review). In this example, comparisons between the two communities are straightforward because the same number of viruses has been enumerated in each. If the number differed, then rarefaction curves could be used to estimate how many taxa would be represented if the larger sample were subsampled to match the size of the smaller one (Gotelli and Colwell, 2001; McCabe, 2011). Alternatively, taxa accumulation curves could be used to estimate how many more species would be gained if the number of individuals enumerated in the smaller sample (Gotelli and Colwell, 2001). For in-depth consideration of such issues, see (Chao et al., 2014).

One must recall that “individual” in this context refers to an individual viral unit, however defined, not to an individual plant, and that “sample-based” assessments include assessments of individual or multiple plants. So with individual-based assessments, for example, one evaluates the number of distinct taxa represented by a given number of virus individuals and then might compare this richness value across treatments. For instance, 100 virus individuals might represent seven taxa in one treatment, and twenty-five in another, giving the latter greater virus richness. One advantage of working with richness values is that taxa accumulation curves and corresponding rarefaction curves may be more directly useful in permitting comparisons. Rarefaction determines how many taxa would likely be present in smaller subsamples of the total sampled population (McCabe, 2011). Thus, a treatment with more individuals can be rarefied to allow more equitable comparison of virus richness with another containing fewer individuals.

### Pooling Strategy

Another crucial parameter is the strategy for pooling individuals or samples for sequencing (e.g., in library preparation), which can be necessary to reduce costs. Individual plants might be pooled, for instance, by species (a subsample of each species present) or by sampling location (all sampled plant species from one quadrat or location). The optimal pool size depends on striking a sometime difficult balance between the number of pools to be sequenced and the number of individual plants per pool. Increasing pool size is likely to exacerbate competition among viruses for sequencing reads; the larger the pool, the higher the probability that some low prevalence or low concentration viruses may be missed if other viruses are present in high abundance (dilution effect). An example is the current practice of inoculating a mild strain of pepino mosaic virus in tomato production to prevent the infection by severe strains. This mild strain is present in high concentration in the plants (up to 25% of total RNA reads, unpublished data). If such plants are included in a pool, the majority of viral reads might come from the PepMV mild strain, hampering the detection of other viruses at low abundance.

This issue is arguably most important in studies that seek to characterize the complete viral community, and perhaps less important for relative comparisons among sampling groups. Nested sample pooling is one approach for determining optimal pooling strategy. In this approach, a series of pools with increasing number of pooled plants from the same community or from an increasing number of communities is collected and sequenced. The results will give a preliminary overview of the geographic heterogeneity of the sampled population and thus of the sample size required for good representation. In all cases, it is advisable to collect and store individual plants for downstream confirmation of HTS results.

Pooling strategies should also consider that some plant species may contain inhibitors (i.e., secondary metabolites) that can negatively affect the amplification and sequencing steps in some protocols (Lacroix et al., 2016). A preliminary study of the potential inhibitory effect of all host species sampled may need to be performed using targeted RT-PCR and mixing experiments (e.g., Lacroix et al., 2016). If inhibition is evident, the preferred solution would be to employ nucleic acid extraction protocols sufficiently robust for all plant hosts sampled. If no other option is available, it may be necessary to exclude the problematic plants species from the study. The dsRNA purification protocol (Tzanetakis and Martin, 2008; Okada et al., 2015; Nwokeoji et al., 2017; Ma et al., 2019) appears to be relatively robust, but in any case, the possibility of limitations for particular plant species should always be considered.

### Selection of Method for Sample Preparation and Sequencing

The selection of the target nucleic acids population is critical as it defines the types of viral sequences that will be detected, including total RNA/DNA, RNA-Seq, Virion-Associated Nucleic Acids (VANA), dsRNA, small RNA, circular ssDNA or amplification of targeted PCR products using generic primers. While HTS technologies have the theoretical capacity to target any viral nucleic acid in any host plant or vector, the available protocols present distinct advantages and limitations as reviewed previously (Roossinck et al., 2015) and summarized in Figure 3 and Table 1.

**FIGURE 3:** Sample preparation for virus ecological studies using HTS. Samples taken from plants, vectors or other sources (waters, animals, etc.) may contain various viral sequences including DNA viruses (blue), RNA viruses (green), viroids (yellow) or viral sequences integrated in the host genome (red). Variants can be produced by mutations (white) and recombinations (black) during the infection. The most frequently used protocols to analyze viral sequences by HTS are based on the extraction of total RNA, dsRNA, small RNA, and Virion-Associated Nucleic Acids (VANA). By using sequencing platforms, sets of reads are obtained and have then to be processed by bioinformatic pipelines to reassemble them in order to detect, identify and quantify the virus and viroids present. Dotted figures correspond to viral sequences sometimes detected with the preparation method described.

**TABLE 1:** Advantages and drawbacks of different sample preparations for HTS-based virus ecological studies.

Nucleic acids	Total RNA	dsRNA	Small RNA (21, 22, 24 nt)	VANA
Advantages	• Detection of any RNA or DNA virus and viroids. • For individual plants and pooled samples.	• All RNA viruses including viroids. • Enrichment of viral sequences in the data. • For individual plants and pooled samples.	• Screen any kind of virus and viroid targeted by silencing mechanism. • For individual plant samples.	• All viral particles, detection of DNA and RNA viruses. • Enrichment of viral sequences in the data. • For individual plants and pooled samples.
Drawbacks	• High sequencing depth is needed as there is a high background of rDNA (even with depletion of ribosomal RNAs). • No enrichment of viral sequences. • Limited sensitivity to detect viruses in low concentration	• Labor intensive. • Limited or no detection of DNA viruses. • Introduction of technical bias (enrichment) for quantification of variants and species.	• Cumbersome extraction methods (Trizol and CTAB-based). • Difficult annotation of sequences and genome reconstruction due to the small size of the sequences. • Only detects actively replicating agents targeted by plant silencing. • Many viruses can have very low sRNA titer in woody crops. • Not yet applied on sample pools for ecological studies. • Complicated assembly requires high sequencing depth in order to be able to assemble and identify viruses. • No enrichment of viral sequences. • Limited sensitivity to detect viruses in low concentration.	• In theory, no detection of viroids or virus nucleic acid not encapsided or with unstable particles. But endornaviruses were demonstrated to be detected with this technique. • Introduction of technical bias (enrichment) for quantification of variants and species. • Highly variable in recovery of viruses.

**The four most frequently used protocols are considered: total RNA, dsRNA, smallRNA, and Virion-Associated Nucleic Acids (VANA) (Cf. Figure 3). Their advantages and drawbacks are presented, in terms of detection, sensitivity, enrichment, convenience, and eventual bias.**

These limitations warrant a careful *a priori* evaluation of the viruses and viroids potentially infecting the plants in the study area. However, neither the viruses, nor their (genomic) characteristics are *a priori* all known. Hence protocol selection may be influenced most strongly by information about which viruses are common in the study area or are most interesting given the question(s) addressed. The research question and the objectives of the study will thus be crucial for protocol selection, along with a botanical inventory. For example, there are currently no viroids known to infect *Poaceae*. So, the VANA method – which concentrates DNA and RNA associated with virions but not viroids – could be a good choice when studying grassland samples, as long as it is understood that the analysis would likely miss any novel *Poaceae*-infecting viroids.

There are additional important considerations in sample and library preparation. For example, many current metagenomics-based protocols include a random PCR amplification step prior to sequencing, which can create chimeric reads and introduce bias in the relative proportion of sequences. This, among others, has so far limited the ability to evaluate the relative frequencies of viral sequences in a sample. Moreover, HTS-based approaches have already proven to be as susceptible to between-samples contamination as PCR-based assays (Massart et al., 2014; Galan et al., 2016), thus requiring specific precautions and controls. These contaminating reads can result from laboratory contaminations but also from read misassignment (also called index-hopping) when multiple libraries that include multiplexed samples are sequenced on the same Illumina lane (Vezzi et al., 2017). In ecogenomic studies where the establishment of a direct link between host plants and virus species is sought, cross-contamination among samples would result in the erroneous identification of virus-host combinations. For example, a plant species might be erroneously identified as a low-titer reservoir for a particular virus. Therefore, the same precautions and standards currently implemented in (RT)-PCR-based assays must be implemented for HTS technologies (Massart et al., 2014; Galan et al., 2016), such as the use of a series of controls (positive/negative, internal/external, spiking) at each step of the HTS pipeline [for example, as developed in the guidelines of the European VALITEST project (Lebas and Massart, 2020)]. In addition, verification of the virus found in individual samples by other independent methods is highly recommended.

In the sequencing phase, proper read length selection is a key consideration. For small RNA sequencing, the very short length of small RNAs (21–24 nt) complicates sequence assembly and annotation, and makes genome reconstruction and strain identification more difficult (Massart et al., 2017, 2019). More typically, read lengths generated by Illumina^TM^ platforms range from 75 to 300 nt for single or paired reads, with error rates increasing with longer reads (Sameith et al., 2016). Pacific Biosciences^TM^ or Oxford Nanopore^TM^ technologies can generate much longer reads (and therefore a better reconstruction of genomes and isolates) but with lower sequencing accuracy (Filloux et al., 2018).

Sequencing depth is directly correlated with an improved ability to detect viruses present at low abundance/concentration, as shown for small RNA sequencing (Massart et al., 2019). On the other hand, a higher sequencing depth increases the probability of false positive detection because of potential contamination problems (i.e., contaminants are more likely to be sequenced) and increases the price per sample (Massart et al., 2014). Protocols allowing an enrichment of viral sequences, such as VANA or dsRNA will significantly improve the sensitivity of virus detection for a given sequencing depth. These protocols are therefore very popular for ecological studies (Djikeng et al., 2009; Coetzee et al., 2010; Blouin et al., 2016; Palanga et al., 2016). On the other hand, total RNA/DNA may still be used despite the requirement of higher sequencing depth (Ng et al., 2011; Bernardo et al., 2013; Gil et al., 2016; Akinyemi et al., 2016). Nevertheless, on the long term, if the cost of sequencing continues to decrease and the efficiency of ribodepletion protocols to increase, the use of total RNA could also be envisioned, provided sufficient sequencing depth is sought (in the range of 100x more than for VANA or dsRNA), as illustrated in grapevine viruses and a 35x enrichment for dsRNA (Al Rwahnih et al., 2009).

### Bioinformatic Analysis

#### Detection, Characterization, and Taxonomic Assignment of Viral Reads and Contigs

Bioinformatic analyses may be performed to examine viral reads and assign them to virus taxonomic units, in order to estimate virus(es) genetic structure and diversity (richness and evenness), or even to characterize novel virus species. However, different population-based or taxonomy-based terms are often used in these analyses, such as virus species, isolates, strains, operational taxonomic unit (OTU) or quasispecies, while their definition has been discussed by virologists (Van Regenmortel, 2007; Adams et al., 2013; Peterson, 2014) and these terms have sometimes been inconsistently used in the literature. The crucial point is thus to define clearly the fundamental unit used for diversity estimation (Claverie et al., 2018). In recent geometagenomics work (Bernardo et al., 2018), virus family was for example defined as the base “individual” unit enumerated to evaluate virus richness per sample, i.e., the number of virus families represented (if any) as determined by BLAST matches of viral contigs. Consequently, this approach was deliberately conservative (to avoid double-counting contigs representing the same viral genome), but could not distinguish and enumerate co-infections of multiple isolates from the same species or of multiples species in the same or in related genera belonging to a family, that can be frequent in nature. Other strategies for estimating the viral diversity from metagenomics-based approaches have been recently used, relying on the use of a clustering of viral conserved protein motifs such as RNA-dependent RNA polymerases (RdRp) to define OTUs representing an acceptable proxy to viral species (Lefebvre et al., 2019; Ma et al., 2019) (see also next section).

Even for a single plant sample, identifying all viral agents present may be a non-trivial bioinformatic challenge and many elements have to be taken into consideration when trying to select a pipeline/strategy and optimize parameters (Massart et al., 2019). The presence of a novel viral species in a sample is not always easily detected and, to some extent, its detection still depends on the expertise of the researcher (Massart et al., 2019). In addition, homology-based annotation approaches, like BLASTn or BLASTx, have limitations because a significant proportion of sequence reads may have no detectable homologs in the sequence databases (Lefebvre et al., 2019) or because some sequences are wrongly annotated databases, which may lead to mis-identifications. Due to these limitations, current virome studies probably still miss part of the viral community but the proportion of viral sequences that are thus unidentified remains a matter of debate. Other approaches like Markov profile (Mistry et al., 2013) or k-mer analyses (Wood et al., 2019) can be used to try to identify novel virus species but without totally solving this issue since their performances are either incomplete or not properly known. Moreover, read assignment can be refined using statistical phylogenetic placement methodology, as recently illustrated by a study focusing on the appropriate phylogenetic position of viral metagenomic reads on a reference phylogenetic *Mastrevirus* tree (Claverie et al., 2019). Beside these homology-based annotation methods, sequence-independent strategies have been developed to identify novel viral sequences without using sequence databases, e.g., through the examination of characteristics of virus-derived small RNAs (Aguiar et al., 2015).

Another crucial issue for taxonomic assignment is the fact that viruses detected in plant samples by HTS technologies may include not only viruses infecting the plant host itself but also those infecting any other organisms caught up in the sample, including microscopic arthropods, bacteria, or fungi living on or in the plant (Shi et al., 2016; Zhang et al., 2019). Some viral taxa may be readily assigned to hosts, on the basis of relationships to existing known viruses. However, the process can be complex if the taxa appear highly novel, are not well accommodated by existing phylogenies, or fall in an intermediate zone of host transition (Dolja et al., 2020; Koonin et al., 2020). Special attention should be paid to the contribution of these “contaminating viruses” to the plant virome, and to the potential influence of sample preparation techniques (e.g., dsRNA isolation might result in overrepresentation of fungal viruses with dsRNA genome as compared to ssRNA plant viruses) (Ma et al., 2019).

The characterization of the biology (host range, transmission mode, symptomatology, geographical distribution, etc.) of any newly identified virus can be challenging too. Indeed, the identification of a putative new virus alone will be of limited usefulness in a range of ecological studies. A characterization framework has recently been published, proposing a scaled approach to progressively and efficiently characterize the biology of a newly identified virus and the associated risks for the wild and domesticated plants (Massart et al., 2017).

#### Viral Richness and Diversity

As discussed, *taxa richness* (the number of taxa present within a sample or environment) and *taxa diversity* (which takes into account both taxa richness and *evenness*, the relative proportions of each taxa) are two key ecological metrics (Whittaker, 1965; Colwell, 1997; Witzany, 2012). To measure richness and diversity from HTS data for viruses is not a trivial task, due to: (i) incomplete virus genome assemblies potentially resulting in different viruses being represented by non-overlapping genome regions (e.g., viral species 1 being represented by its capsid protein gene while viral species 2 is represented by it polymerase gene); (ii) chimeric assembly due to homologous regions as explained in “Co-infection by Several Viruses”; and (iii) the challenge of defining enurable viral units (see above). Non-homogeneous taxonomic criteria between viral families and the absence of universally conserved genomic region shared by all viruses further complicate viral richness estimation. This difficulty will also impact alpha, beta or gamma diversity analyses, with the added complexity of simultaneously necessitating quantitative abundance or prevalence data for each individual agent (see section on “Infection Prevalence”).

A proposed strategy is to measure a proxy of virus species richness by enumerating OTUs. This can be achieved by aligning a conserved region, often part of the polymerase region, setting an arbitrary distance separating OTUs (more than a fixed percentage of divergence) and then performing a sequence clustering. Other proxys have been used to estimate viral richness, for example the number of viral families or genera, or OTUs defined using other approaches but these other proxys tend to have even more limitations than the use of OTUs based on a clustering approach. A very good description of this approach for virus classification was presented by Simmonds (2015). It has recently been implemented in at least one annotation pipeline (Lefebvre et al., 2019), and already used at the family level in ecological analyses combined to plant spatial distribution (Bernardo et al., 2018) and near species level for the benchmarking of sequencing strategies (Ma et al., 2019). The study of taxa richness based on similarities/divergence between sequences offers the possibility to taxonomically “assign” the large number of virus sequences generated by HTS, but also presents some pitfalls. Indeed, while numerous virus genomes have experienced recombination and reassortment event(s), only complete genomes or at least complete coding regions of virus genomes are suitable for reliable taxonomic assignments (Simmonds, 2015). However, despite these limitations to precise taxonomic assignment, distance-based methods can be used as the only source of information for virus richness estimation from HTS data.

#### Single-Nucleotide Polymorphisms (SNPs) and Virus Populations

Viral populations can evolve quickly by mutation and/or recombination at each replication cycle. The resulting variants may bear large genome rearrangements as well as single-nucleotide polymorphism (SNP) mutations. Accessing viral intra-specific diversity through HTS has value for specific scientific aims (Beerenwinkel and Zagordi, 2011), such as to better measure and map evolutionary footprints of virus emergence at the plant community scale. For example, the detailed characterization of viral isolates will be needed in order to compare the virus population in a primary host and in potential reservoir(s).

To genotype and haplotype SNPs remains a challenging bioinformatic task for a single virus in a single sample. It becomes obviously more complex with samples containing multiple viruses from multiple hosts. In the case of mixtures of isolates, reconstruction of genomic sequences may be particularly complex, if not altogether impossible, especially when multiple closely related isolates are involved or for quasi-species with high variability. Moreover, the differentiation between SNP and sequencing errors is intrinsically difficult for low frequency variants. It can be impacted by the quality of the HTS sequences produced, by read length, but also by the algorithms used for quality control, contig assembly, and SNP identification. The statistical approach selected for the haplotyping analysis is another key factor to consider; its performance is determined by mutation rate and was demonstrated to decrease with genetic diversity of the sample (see McCrone and Lauring, 2016; Posada-Cespedes and Seifert, 2017; Eliseev et al., 2020).

The confirmation of SNPs represents another challenge: targeted real-time PCR could be used but the need to design and produce two probes per SNP remains costly. Another potential way to reinforce the significance of the analysis is to sequence duplicates of each sample or to combine the use of different HTS approaches that have different distribution of sequencing errors. While costly, these approaches have the potential to distinguish true SNPs from sequencing errors. Running duplicates is a strategy that is often performed for HTS-based barcoding (Razzauti et al., 2015) and could be applied to virus ecology.

## Conclusion

The study of plant virus ecology, which began at the end of the 19th century, has been accelerated by the evolution of new methods used to detect plant viruses in various environments and in many plants simultaneously: the HTS technologies offer huge opportunities to improve virome characterization and address novel questions such as the examination of virus spread among host reservoirs (wild and domestic), the effects of ecosystem simplification caused by human activities (and agriculture) on the biodiversity, and the emergence of new viruses in crops. Recently, conceptual shifts in the understanding of the origins and diversification of the plant virome were achieved, leading to the design of the first comprehensive virus megataxonomy. Nevertheless, the use of HTS in ecological studies is associated with a series of challenges and pitfalls described in detail in this review for each procedural step in the field, in the laboratory and for bioinformatic analyses. The rapid evolution of the sequencing platforms and bioinformatic pipelines promises numerous findings in viral metagenomic studies over the coming years. These novel approaches developed in plant virology will directly be transferable to other models for a better understanding of host-virus interactions and ecological virology in general.

## Author Contributions

FM and SM conceived and wrote the manuscript. FM created the figures and prepared the final version of the manuscript and all authors approved it. In particular, PR and CM edited the viromics advances and field sampling sections, respectively. TC, CM, PR, RV, and DF edited the bioinformatics sections. All authors collectively revised and improved the manuscript and made useful suggestions on all sections of the review article.

## Conflict of Interest

The authors declare that the research was conducted in the absence of any commercial or financial relationships that could be construed as a potential conflict of interest.

## Footnotes

1 https://digitalcommons.unl.edu/cgi/viewcontent.cgi?article=1016&context=usblmpub
